# Correlation of IgH-CDR3 Immune Repertoire Diversity Test in Peripheral Blood of Neuromyelitis Spectrum Diseases

This article has been retracted.

**DOI:** 10.1155/2022/6790145

**Published:** 2022-10-10

**Authors:** Zhihui Peng, Hongfei Deng

**Affiliations:** ^1^Internal Neurology, Shaoyang University Affiliated Second Hospital, Shaoyang, 422000 Hunan, China; ^2^Precision Medicine Center, First People's Hospital, Chenzhou, 423000 Hunan, China

## Abstract

Neuroretinitis spectrum disorder (NMOSD) is generally regarded as an acute or subacute inflammatory demyelinating disease of the central nervous system, mainly involving the optic nerve and spinal cord, mediated by humoral immunity. To address these questions, this work established an immunomic library of the heavy chain complementarity determinant 3 (gHI-CDR3) of peripheral blood lymphocyte B cell receptors. The library was established in patients with a spectrum of neurosyphilis-retinitis disorders. Six NMOSD patients and six healthy volunteers were recruited, and the NMOSD group was divided into an early-onset group and a stable group according to treatment conditions. The IgH-CDR3 gene fragment cultured in vitro was amplified by multiplex PCR technology, and the gene was sequenced by the second-generation high-throughput sequencing technology, and the statistical analysis was carried out by the method without reference. The quantity, type, and diversity of IgH-CDR3 in peripheral blood B lymphocytes of NMOSD patients were significantly lower than those of normal group (*P* > 0.05); the variation of IgH-CDR3 sequence in the initial stage of treatment was higher than that in the stable stage (*P* > 0.05); the replication frequency of the characteristic gene “CASSICLGSGCGGYYYGMDVW” was significantly increased in patients at the initial stage of NMOSD treatment (*P* < 0.05). The conclusion was that the gene expression and gene expression analysis of NMOSD patients could accurately judge the condition of NMOSD patients, evaluate their efficacy, and provide new molecular targets and new theoretical basis for clinical application.

## 1. Introduction

Neuropathic blepharitis spectrum disorder (NMOSD) is a major disease of the CNS caused by self-generated immune response, mainly in the optic nerve, spinal cord, and other parts as the main symptoms. Conventional gene sequence detection methods are mainly based on Sanger sequences or gene sequences, but their clinical application is greatly restricted due to technical shortcomings such as low resolution and low throughput. With the continuous development of high-quality quantitative technology, vaccination technology has developed rapidly, reducing the time and cost of vaccination and improving the effectiveness of vaccination. The disease has a high incidence in non-Caucasian regions and is more common in young people, women, and relapses. The morbidity rate and mortality rate are high, so its prognosis is generally poor; the pathogenesis of NMOSD needs to be further explored, among which humoral immunity with B lymphocytes as the carrier is the main research direction. Further understanding of the role of the B lymphatic system will help improve the efficacy and individualization of NMOSD and facilitate the diagnosis and treatment of NMOSD.

CNMOSD is mainly a recurrent inflammatory disease of the CNS. Oertel et al.'s study showed that the use of OCT could detect not only damage to the afferent visual system caused by ON but also NMOSD-specific intraretinal lesions, astrocytopathies [1]. A controlled study by Xie et al. assessed this association by recruiting 305 patients with neuromyelitis optica spectrum disorder and 487 healthy controls in a neurology department. Peripheral blood was collected, DNA was extracted, and GTF2IRD1-GTF2I polymorphism was analyzed by genotyping for neuromyelitis optica spectrum disorder in Chinese Han population. The results indicated that the T allele was associated with an increased risk of neuromyelitis [2]. MR imaging and optical coherence tomography are essential in the diagnosis and evaluation of NMOSD. Akaishi et al. studied the clinical and MR imaging findings of anti-aquaporin-4 antibody-seropositive and anti-myelin oligodendrocyte glycoprotein antibody-seropositive NMOSD [3]. The aim of the Lersy et al. study was to highlight cervical spinal cord atrophy in NMO patients compared with controls and to assess the correlation between atrophy and clinical features and cervical spinal cord MRI data. His study investigated 15 patients diagnosed with NMOSD and 15 healthy patient controls. The results showed that the mean CSA was 68.5 mm^2^ in the NMO patient population and 72.8 mm^2^ in the healthy subject population [4]. The Paton study showed that NMOSD was a rare autoimmune disorder in which patients experienced relapses affecting the optic nerve, spinal cord, or brainstem. NMOSD was more common in women, with onset around the age of 30-40 years, depending on ethnicity [5]. However, these studies did not conduct a corresponding correlation study on the diversity test of the IgH-CDR3 immune repertoire.

Correlation studies on the diversity test of the IgH-CDR3 immune repertoire in peripheral blood of NMOSD have become crucial. Gao et al. reviewed the pharmacological profile, clinical evidence, and therapeutic status of satralizumab in the treatment of NMOSD. A phase III trial demonstrated a protocol-defined recurrence rate of 30% when patients with NMOSD received satralizumab monotherapy, compared with 50% in the placebo group (*P* = 0.018), and a protocol-defined recurrence rate of 20% for satralizumab [6]. The purpose of Sm A was to assess the prevalence and diagnostic value of anti-AQP4 antibodies in Tunisian patients with such inflammatory neurological diseases. The diagnosis of NMOSD was made in 7 seropositive patients and 2 seronegative patients by testing for anti-AQP4 antibodies in 170 consecutive Tunisian patients with inflammatory disease of the central nervous system and optic cord involvement. This resulted in a seroprevalence of 77.7% in the NMOSD subgroup [7]. Li et al.'s studies found that during NMOSD, microglia could be activated by interleukin- (IL-) 6 and type I interferons (IFN-Is), leading to signal transducer and activator of transcription (STAT) activation. They studied the latest research progress on the role of microglia in the pathogenesis of NMOSD, the mechanisms of microglia activation and microglia-mediated inflammation, and potential research prospects [8]. Research by Baghbanian et al. showed that autoantibodies to the aquaporin 4 (AQP4) caused humoral inflammatory demyelination and axonal damage [9]. Zhang et al. collected data on 40 patients with CTD LETM admitted to the Department of Neurology or Rheumatology, divided into two groups: CTD-LETM-NMOSD and CTD-LETM-non-NMOSD. The Kaplan-Meier method was used to analyze the recurrence rate and clinical outcome [10]. However, the limitations of technical methods largely limit the development of immune repertoire research. Commonly used immune repertoire sequencing technologies include PCR technology, immune scanning lineage analysis technology, and flow cytometry. Although these techniques have their own characteristics, there are also obvious deficiencies, such as a small amount of effective information and a large number of influencing factors.

The frequency distribution of IGHV3-23 in peripheral blood B cells in the NMOSD group at baseline was 0.083 + 0.014, which was higher than that in the healthy people, 0.062 + 0.015. Compared with healthy controls, the stability group was significantly higher by 0.062-0.015; The polymorphisms of HI-CDR3 gene in peripheral blood of patients in group 3 (NMOSD) and non-NMOSD (2, 3) groups were 3.33 (*n* = 0.71) and 4.30 (*n* = 0.29) (*n* = 6), respectively.

The innovation of this paper is that the biggest problem in the analysis of the gene sequence of the immune group is the introduction of the gene sequence. Arm-PCR technology can accurately reflect the ratio of each clone and ensure the solubility of each CDR3 gene. Using arm-PCR technology for high-quality, large-sample sequence analysis of NMOSD patients can better understand the pathogenesis of NMOSD, thereby laying the foundation for discovering the disease state of NMOSD, monitoring efficacy, and immunotherapy. By using the next-generation high-throughput sequencing technology and multiplex PCR technology, the most abundant CDR3 region of BCR in the peripheral blood of NMOSD patients is amplified, and the related gene library of IgH-CDR3 is obtained. On this basis, the characteristics of the antibody library at each stage are compared and compared with clinical data.

## 2. NMOSD Peripheral Blood IgH-CDR3 Immune Repertoire Diversity Method

### 2.1. Etiology and Immune Pathogenic Mechanism of NMOSD

NMOSD is caused by genetic factors, and its onset and recurrence vary geographically and seasonally. 90% of non-MOSD patients have a certain relationship with HLA alleles of DRB1∗0501 and DRB1∗0301 alleles. DRB1∗0301 is the most prevalent in Caucasian populations, while non-Asian populations are responsible for DRB1∗0501 [11]. In blood-brain protection, AQP4 has specific connection with AQP4 receptor, thus affecting the distribution of AQP4 on its surface. This will enhance the permeability of the blood-brain barrier, make the edema and inflammatory cells around the blood vessels infiltrate, and enhance the permeability of the body's immunity and antibodies through the blood-brain barrier, thereby making the body's immune function more serious [12]. NMOSD is a very complex immune system, which includes the immune regulation disorder of the immune system, including humoral immunity, T lymphocyte mediated immunity, immune cell mediated immunity, immune cells (e.g., macrophages and hemophagocytic cells), and immune cells such as cytokines. The in-depth discussion of the immune mechanism of NMOSD has laid a theoretical basis for the clinical application of NMOSD.

### 2.2. Role of Cells in the Pathogenesis of NMOSD

The etiology of NMOSD is unknown, but a large number of clinical and basic experimental results show that B cells are involved in the occurrence of NMOSD. About 75% of NMOSD patients will produce autoimmune water vapor 4 (AQP4), as well as other kinds of autoantibodies [13]. This causes inflammation and demyelination. However, in practical applications, the immune response of AQP4 has nothing to do with the active degree and recurrence of the disease, and the AQP4 antibody does not significantly decrease after alleviation, suggesting that the occurrence of NMOSD does not depend solely on the production of AQP4. In recent years, a large number of clinical data have shown that the abnormality of the B lymphatic system is related to the occurrence of NMOSD [14].

### 2.3. Sequencing Technology of Immune Repertoire

The technology can not only detect T lymphocytes but also can analyze the function of T lymphocytes and lay a foundation for clinical diagnosis, treatment, and clinical application. This method can only perform preliminary analysis on CDR3 variants or certain sequences, and further research is required at the genetic level to better understand how CDR3 differs from disease behavior, pathogenesis, and the normal human immune system. As a representative of “next-generation” sequence (NGS) technology, 454 SOLiD sequence, and HiSeq gene detection platform (HiSeq) technology, it has comprehensively demonstrated the status of vaccines [15]. By uploading the sequence information of the original sequence to the sequences of each sample, the redundant sequences, short fragments, and sequences with lower sequences in these sequences were compared and searched by iRmap technology, and the CDR3 peptide chain sequences of each sample were compared and searched [16]. The samples were analyzed by two-dimensional heat map, D50, and other methods. By using CDR3 list, D50, dendrogram, V distribution, CDR3 length distribution, N-terminal added base number distribution, and other indicators and graphics, the immune characteristics of the samples were studied.

### 2.4. Deep Learning Algorithms

Deep learning can be seen as a collection of neural network models. What these models have in common is an input layer, an output layer, and several hidden layers [17]. The structure of a single neuron is shown in Figure 1.

As shown in Figure 1, a weighted sum of the input signal is obtained, and a nonlinear mapping is performed as the output of the neuron.

(1) $$\begin{array}{c} b=f\left(\overset{K}{\underset{i=1}{\sum }}w_{i}a_{i}\right)=f\left(W^{T}A\right). \end{array}$$

The role of the nonlinear function is to restrict the output in the range of 0 to 1 through nonlinear mapping, which is also commonly referred to as the excitation function [18]. Taking the sigmoid function as an example, the output of the neuron is shown in

(2) $$\begin{array}{c} b=\frac{1}{1+e^{W^{T}A}}. \end{array}$$

The purpose of deep learning is to learn the features of the input data so that the output *b* of the network and the target output *b*_target_ are as close as possible [19]. The loss function can be defined as shown in

(3) $$\begin{array}{c} Q=\frac{1}{2}{\left(b_{\text{target}}-b\right)}^{2}=\frac{1}{2}{\left(b_{\text{target}}-f\left(W^{T}A\right)\right)}^{2}. \end{array}$$

The gradient of the loss function with respect to the specified weight *W*_*i*_ can be expressed as shown in

(4) $$\begin{array}{c} \frac{\partial Q}{\partial w_{i}}=\frac{\partial Q}{\partial b}\cdot \frac{\partial b}{\partial u}\cdot \frac{\partial u}{\partial w_{i}}=\left(b-b_{\text{target}}\right)\cdot b\left(1-b\right)\cdot a_{i}. \end{array}$$

According to the most subduction algorithm, each variable is in the form of a vector, and the repetition of the weight is shown in

(5) $$\begin{array}{c} w^{\text{new}}=w^{\text{old}}-\mu \cdot \left(b-b_{\text{target}}\cdot b\left(1-b\right)\cdot a\right), \end{array}$$

where *μ* > 0 is the step size of gradient descent, which determines the size of weight decay in each iteration [20]. The simplest neural network structure is shown in Figure 2.

As shown in Figure 2, the input layer contains *X* neural units, denoted as *A* = {*a*_1_, *a*_2_, ⋯, *a*_*x*_, }; the hidden layer contains *Y* neural units, denoted as *g* = {*g*_1_, *g*_2_, ⋯, *g*_*y*_}; the output layer contains *K* neural units, denoted as *b* = {*b*_1_, *b*_2_, ⋯, *b*_*k*_} [21]. The output of a single hidden unit can be expressed as

(6) $$\begin{array}{c} g_{y}=f\left(u_{y}\right)=f\left(\overset{N}{\underset{x=1}{\sum }}W_{xy}a_{x}\right). \end{array}$$

The output of a single output unit can be expressed as shown in

(7) $$\begin{array}{c} b_{k}=f\left(u_{k}^{\prime }\right)=f\left(\overset{Y}{\underset{y=1}{\sum }}W_{yk}^{\prime }g_{y}\right). \end{array}$$

At this time, the loss function of the entire neural network is shown in

(8) $$\begin{array}{c} Q=\frac{1}{2}\overset{K}{\underset{k=1}{\sum }}{\left(b_{k}-b_{{\text{target}}_{\text{k}}}\right)}^{2}. \end{array}$$

Unlike the training of a single neuron, the training of a neural network needs to update both the *w*_*ij*_ stage and the *w*_*ij*_′ stage, so it is necessary to calculate the bias function of the loss function of the two weights [22]. At the same time, an update is performed. According to the chain law, the partial derivative function of the loss function related to the *w*_*ij*_′ phase is shown in

(9) $$\begin{array}{c} \frac{\partial Q}{\partial w_{ij}^{\prime }}=\frac{\partial Q}{\partial b_{j}}\cdot \frac{\partial b_{j}}{\partial u_{j}}\cdot \frac{\partial u_{j}}{\partial w_{ij}^{\prime }}, \end{array}$$

where

(10) $$\begin{array}{c} \frac{\partial Q}{\partial b_{j}}=b_{j}-b_{{\text{target}}_{\text{j}}}, \end{array}$$

(11) $$\begin{array}{c} \frac{\partial b_{j}}{\partial u_{j}^{\prime }}=\frac{\partial f\left(u_{j}^{\prime }\right)}{\partial u_{j}^{\prime }}=f\left(u_{j}^{\prime }\right)\left(1-f\left(u_{j}^{\prime }\right)\right)=b_{j}\left(1-b_{j}\right), \end{array}$$

(12) $$\begin{array}{c} \frac{\partial u_{j}^{\prime }}{\partial w_{ij}^{\prime }}=\frac{\partial \left(\sum_{y=1}^{Y}W_{yj}^{\prime }g_{y}\right)}{\partial w_{ij}^{\prime }}=g_{j}. \end{array}$$

The original formula (9) can be simplified as

(13) $$\begin{array}{c} \frac{\partial Q}{\partial w_{ij}^{\prime }}=\left(b_{j}-b_{{\text{target}}_{j}}\right)\cdot b_{j}\left(1-b_{j}\right)\cdot g_{i}. \end{array}$$

Then, the update formula of *w*_*ij*_′ can be expressed as

(14) $$\begin{array}{c} {w^{\prime }}_{ij}^{\text{new}}={w^{\prime }}_{ij}^{\text{old}}-\mu \cdot \left(b_{i}-b_{{\text{target}}_{j}}\right)\cdot b_{j}\left(1-b_{j}\right)\cdot g_{i}. \end{array}$$

Next, the weight update method for input units and hidden layer units is discussed [23]. In addition, according to the chain law, the partial derivative function of the loss function related to *w*_*ij*_ is shown in

(15) $$\begin{array}{c} \frac{\partial Q}{\partial w_{ij}}=\frac{\partial Q}{\partial g_{j}}\cdot \frac{\partial g_{j}}{\partial u_{j}}\cdot \frac{\partial u_{j}}{\partial w_{ij}}=\left(\overset{K}{\underset{k=1}{\sum }}\frac{\partial Q}{\partial b_{k}}\cdot \frac{\partial b_{k}}{\partial u_{k}^{\prime }}\cdot \frac{\partial^{\prime }u_{k}}{\partial g_{j}}\right)\cdot \frac{\partial g_{j}}{\partial u_{j}}\cdot \frac{\partial u_{j}}{\partial w_{ij}}. \end{array}$$

The partial derivative formula is more complicated than formula (15), because the weight *w*_*ij*_ is actually associated with each output unit [24].

(16) $$\begin{array}{c} \frac{\partial u_{k}^{\prime }}{\partial g_{j}}=\frac{\partial \left(\sum_{y=1}^{M}W_{yk}^{\prime }g_{y}\right)}{\partial g_{j}}=W_{jk}^{\prime },\\ \frac{\partial g}{\partial u_{i}}=g_{j}\left(1-g_{j}\right),\\ \frac{\partial u_{j}}{\partial w_{j}}=\frac{\partial \left(\sum_{x=1}^{X}W_{xj}^{\prime }A_{x}\right)}{\partial w_{ij}}=X_{i}. \end{array}$$

From formulas (10) and (11), it can be known that

(17) $$\begin{array}{c} \frac{\partial Q}{\partial b_{k}}\cdot \frac{\partial b_{k}}{\partial u_{k}^{\prime }}=\left(b_{k}-b_{{\text{target}}_{k}}\right)\cdot b_{k}\left(1-b_{k}\right). \end{array}$$

Formula (15) can be simplified as

(18) $$\begin{array}{c} w_{ij}^{\text{new}}=w_{ij}^{\text{old}}-\mu \cdot \overset{K}{\underset{k=1}{\sum }}\left[\left(b_{k}-b_{{\text{target}}_{k}}\right)\cdot b_{k}\left(1-b_{k}\right)\cdot w_{jk}^{\prime }\right]\cdot g_{j}\left(1-g_{j}\right)\cdot a_{i}. \end{array}$$

## 3. Correlation Experiments for Diversity Test

### 3.1. Materials and Methods

A total of 6 NMOSD patients were included in this trial, who were admitted to the hospital or outpatient clinic from May 2015 to December 2017 and were divided into two periods: initial and late stable.

Eligibility criteria are as follows: all selected patients met the international standards of NMOSD in 2015, AQP4-IgG was negative, standardized treatment was performed within more than one month of onset, 18 to 65 years of age, no pregnancy on follow-up, follow-up of more than 8 months, and no recent symptoms.

Exclusions are as follows: other inflammatory demyelinating lesions, such as multiple sclerosis, demyelinating pseudotumor and acute disseminated encephalomyelitis; recent infections such as urinary tract infection, acute respiratory infection, and digestive system infection; infectious diseases associated with immunodeficiency, such as immunodeficiency and AIDS; long-term use of immunosuppressants; recent viruses; and have been vaccinated recently.

There were NMOSD 6 women aged 31 to 47, 6 of whom were AQP4 antibody negative; 3 patients had initial NMOSD; 3 patients did not have it; 2 patients had optic nerve signs first, 2 patients had spinal signs, and 2 patients had optic nerve signs and spinal signs. Two patients received 1000 mg of the drug, two received 1000 mg of hormone, two received 500 mg of hormone, two received 80 mg of hormone, and two received additional glucocorticoids. Specimens were collected 1 month after the operation and more than 8 months after the operation. Six healthy female volunteers were selected and compared by gender and age.

### 3.2. Correlation Experiment Process of Diversity Test

*Data collection*: all cases were recorded in detail by specialist physicians and received corresponding auxiliary diagnosis. There is routine examination of blood, urine, feces, liver, and kidney function. Brain and/or spine MRI images, AQP4 antibodies, EDSS score, B-lymphocyte ratio, and treatment of choice.

*Blood samples*: in the morning, all subjects took 2 ml of blood on an empty stomach and left it for 15 minutes after sampling. After 10 min of centrifugation at 3000 rpm, the supernatant was collected and placed in a centrifuge test tube at -80°C for testing. This prevented repeated freezing of samples, which can cause damage to the samples.

*Technical steps*: multiplex PCR technology was used to amplify CDR3 in BCR. The steps were as follows: (1) the volume of the DNA sample was obtained from the sample test results with a starting DNA amount of 400 ng. (2) This sample was subjected to multiple PCRs with specially designed primers containing the V fragment of the Illumina region and the primers of the J region. (3) The compound PCR product was purified by 1 times the capacity of Agencourt AMPure XP microspheres. (4) The purified DNA was fragmented with Agencourt AMPure XP magnetic beads. (5) Secondary amplification was performed using the primers of the Illumina flow cell gene. (6) The PCR product was cut into target size fragments by agarose gel electrophoresis, then colloidally purified with QIAquick Gel Extraction Kit, then dissolved in elution buffer, and then marked with the book collection logo, thus realizing the construction of the library. (7) Library quality management: Agilent 2100 Bioanalyzer was used to detect the debris of the database; ABI StepOne P1us Real-Time PCR system (TaqMan Probe) was used to quantify the density of the database. (8) Illumina's test platform is used for sorting. The checked library was made monomolecular by addition of NaOH, diluted to a specific concentration at the desired loading density, and the denatured sparse library was added to the flow cell. Flow cell hybridization was performed with flow cell, bridge PCR was performed on the cBot cluster generation platform, and finally, the sequence of PE151 was determined.

*Data processing*: MiXCR's antibody library sequencing software was used to sequence along with the gene library. The same series is the same clone. To reduce errors from PCR and sequencing, low-quality data were compared twice. The result was a table-separated text file, each containing the clone class number, frequency, CDR3 sequences, V/D/J genes, etc. Based on these data, further research was carried out. The main contents include CDR3 length distribution, V/J gene usage frequency, V/J combination frequency, sequencing saturation curve, cloning frequency distribution, diversity index, multisample cocloning, hierarchical clustering, and MDS clustering.

### 3.3. Correlation of NMOSD Diversity Test

In this study, the Hiseq4000 platform was used to perform immunomic sequencing on the samples submitted for inspection, and the peripheral blood IgH-CDR3 immunomic library information was obtained from 6 early-stage stable NMOSD patients and 6 healthy volunteers, with a total of 18 samples. The basic information of the immune repertoire of the research specimens is shown in Table 1.

As can be seen from Figure 1, in early and stable NMOSD patients, the total number and species of IgH-CDR3 were lower than those in normal controls. Compared with other patients and healthy controls, the type of peripheral blood IgH-CDR3 and the ratio of CDR3 type to peripheral blood CDR3 were significantly increased in the early stage of treatment.

In the NMOSD patient group, the amino acid sequence length of IgH-CDR3 extracellular B lymphocytes was basically the same as that of the healthy controls, but the amino acid sequence lengths were significantly different in different ranges. In peripheral blood B lymphocytes, the amino acid sequence of LgH-CDR3 gene could be seen.

As can be seen from Figure 3, the gene fragment of IgHI-CDR3 had 4-50 amino acids (aa) in both NMOSD patients and healthy controls and was distributed close to normal. In NMOSD patients, the amino acid sequence of the IgH-CDR3 region was less frequently expressed between 12-14 aa and 16-18 aa; in NMOSD patients, the expression of gene sequences in the IgHI-CDR3 region between 21 and 29 aa was less than in normal subjects.

#### 3.3.1. Frequency of Use of V Gene and J Gene

IGHJ 1, IGHJ2, IgHJ3, and IGHJ4 subgroups were significantly higher than those in the normal control group before and after treatment, while the frequency of subfamily was significantly lower than that in the normal control group. The frequency distributions of TOP20-V and J-type are shown in Figure 4.

As can be seen from Figure 4(a), the application frequency of IGHV3-30 in peripheral blood B lymphocytes was0.078 + 0.026(*n* = 6) and 0.081 + 0.027(*n* = 6), respectively. There were no significant differences among them. As shown in Figure 4(b), the application frequency of IGHJ5 in the stable group was 0.077 + 0.02 (*n* = 6), which was significantly higher than that in the peripheral blood of the healthy control group. The application frequency of B lymphocyte IGHJ5 was 0.124 × 0.009 (*n* = 6).

#### 3.3.2. Diversity Analysis of Immune Repertoire

In this study, the diversity of the peripheral blood IgH-CDR3 B cell immune system repertoire in the NMOSD patient group showed a downward trend compared with the diversity of the IgH-CDR3 B cell immune system repertoire in the control group. In this study, the D50 index, which was newly introduced in recent years to represent the structure of the sample clone population, was used as the evaluation index of IgH-CDR3 sequence diversity. The statistical table of the clone diversity index is shown in Table 2.

As can be seen from Table 2, compared with the D50 of the normal control group, the IgH-CDR3 sequence diversity of peripheral blood B cells in the early treatment group was 4.08 ± 1.21 (*n* = 6). The stable NMOSD group was 3.13 ± 1.35 (*n* = 6), both lower than the normal control group's 4.30 ± 0.29 (*n* = 6), but the difference was not statistically significant. The diversity of IgH-CDR3 sequences in peripheral blood of NMOSD patients was higher in the early treatment group than in the stable group (except for patient number). D50 and D50 were 4.42 ± 1.04 (*n* = 5) and 2.82 ± 1.27 (*n* = 5), respectively, but the difference was not statistically significant; the D50 diversity of IgH-CDR3 genes in peripheral blood in the early stage of NMOSD (except patient 3) was 3.33 + 0.71 (*n* = 4) and 4.30 + 0.29 (*n* = 6). The expression of IgH-CDR3 gene in peripheral blood B lymphocytes of NMOSD (NMOSD) stable group was also significantly decreased, with D50 of 2.82 + 1.42 (*n* = 5), which was significant compared with the control group (*P* < 0.05). On the basis, the D50 value of patients 2 and 3 was 5.93, while the D50 value of normal subjects was significantly higher.

#### 3.3.3. Screening and Analysis of Disease-Predominant Sequences

The NMOSD gene was initially screened and verified. In this paper, the IgH-CDR3 gene sequences of 6 cases of NMOSD and 6 cases of healthy people were compared, and the expression levels of IgH-CDR3 genes were compared (considered significant). The gene expression of lgH-CDR3 had good significance in the two NMOSD patients who received combined stable therapy in the two early stages of NMOSD. NMOSD patients had 2,302 gene fragments on the B cell membrane at the beginning of treatment. In patients with early NMOSD, a total of 2302 IgH-CDR3 genes were found, of which 1723 genes were expressed on the B cell membrane of NMOSD patients. A total of 279 genes were found in 5 early-stage NMOSD patients, while 238 genotypes were stable genes in 5 NMOSD patients. The IgH-CDR3 sequence library of peripheral blood B lymphocytes of NMOSD patients was compared with that of healthy controls, and on this basis, two gene fragments with specific pathogenic characteristics, “CASSICLGSGCGGYYYGMDVw” and “CARPNYYGSVRTGYGMDVWw,” were selected. The predominant lgH-CDR3 sequences of the 2 NMOSD patients in the early stage of combined stable therapy are shown in Tables 3 and 4.

As can be seen from Tables 3 and 4, the gene cloning frequency of “CASSICLGSGGcGYYYGMDVW” was significantly higher in the patients with NMOSD than those of the former NMOSD, with a cumulative number of 21,429. In 2 patients, the number of repeats of this gene was 6, as can be seen from Tables 3 and 4. However, in the B sequence library of the IgH-CDR3 gene of NMOSD patients, the cumulative number of occurrences of this gene is only 3229, and the patient's gene expression rate is 6; similarly, in the gene pool of IgH-CDR3 subgroup, the expression frequency of IgH-CDR3 gene is only 3477.

In this study, although a decrease in the total number of IgH-CDR3 and CDR3 species in peripheral blood B cell subsets in 6 NMOSD patients could be observed compared to normal controls, the difference was not statistically significant. Moreover, the distribution of IgHI-CDR3 amino acid sequence length in the peripheral blood of NMOSD patients in the early stage and in the stable stage showed an approximate normal distribution. This result was consistent with the control group, indicating that there was no overall shift in the number and type of IGHI-CDR3 in peripheral blood B cells of NMOSD patients. But interestingly, the total number of IgH-CDR3, CDR3 types, and diversity index of D50 immunohistochemical repertoire in peripheral blood of patients 2 and 3 were significantly higher than those of other NMOSD patients and normal controls. Notably, these two patients received 100 mg after the start of pulse hormone therapy, while the other patients received only 500 mg or less after the start of pulse hormone therapy. This showed that the immune systems of these two patients were relatively active in the early stages of treatment, and it can be speculated that high-dose hormone pulse therapy mobilized the immune systems of NMOSD patients and significantly increased the diversity of the immune repertoire in a short period of time.

### 3.4. ROC Curve of ReHo Signal

The ROC curve was used to analyze the diagnostic value of ReHo signal for abnormal brain regions. The ROC curve analysis of the Rello signal in AQP4-positive patients and healthy controls is shown in Figure 5.

As shown in Figure 5(a), AQP4-positive patients had increased Relo signal in the left inferior frontal gyrus compared with healthy subjects, AUC = 0.78 (*P* = 0.002; 95%, CI. 0.639-0.921); as shown in Figure 5(b), AQP4-positive patients had decreased Relo signal in the right middle temporal gyrus/occipital gyrus compared with healthy controls, AUC = 0.795 (*P* < 0.001; 95%, CI: 0.658-0.932). The ROC curve analysis of the Relo signal in the anti-MOG antibody-positive patients compared with the healthy control group is shown in Figure 6.

As shown in Figure 6(a), the ReHo signal in the left posterior lobe of the brain in the MOG-positive patients was reduced compared with that in the healthy subjects, AUC = 0.884 (*P* < 0.001; 95% CI: 0.658-0.932); as shown in Figure 6(b), the Reo signal in the left inferior frontal gyrus was increased in MOG-positive patients compared with healthy subjects. The ReHo signal in the right middle-anterior gyrus increased, ALC = 0.869, and the ReHo signal in the left middle-anterior/middle-posterior gyrus increased, AUC = 0.872. The ROC curve analysis of Relo signal in AQP4-positive patients compared with healthy controls is shown in Figure 7.

As shown in Figure 7(a), the ReHo signal in the right posterior cerebellar lobe of MOG-positive patients was reduced, with AUC = 0.835; as shown in Figure 7(b), the ReHo signal in the left middle anterior/middle posterior gyrus increased, AUC = 0.913; the ReHo signal in the right superior temporal gyrus increased, AUC = 0.935.  Figure 8 shows the correlation analysis between serum IL-36 levels and clinical characteristics in NMOSD patients.

As shown in Figure 8, the levels of IL-36*α* and IL-36*β* in serum were not associated with the annual recurrence rate of all NMOSD patients, whereas IL-36*γ* was positively correlated with the annual recurrence rate of NMOSD patients. The higher the level of IL-36*γ*, the greater the patient's annual recurrence rate.  Figure 9 shows the correlation between serum IL-36 levels and the number of affected spinal cord segments.

As shown in Figure 9, serum levels of IL-36*α*, IL-36*β*, and IL-36*γ* did not correlate with the number of affected spinal cord segments in NMOSD patients. The correlation analysis between serum IL-36 level and EDSS score is shown in Figure 10.

As shown in Figure 10, serum levels of IL-36*α*, IL-36*β*, and IL-36*γ* did not correlate with EDSS scores in NMOSD patients.

## 4. Conclusions

When studying disease-specific biomarkers, high-throughput sequencing can be used to find disease-specific CDR3s in patients with the same disease, and these CDR3 sequences are then used as a proxy for the disease. These validated CDR3 sequences can then be used as disease biomarkers and can be identified in peripheral blood; individuals in subhealth or disease states have reduced levels of immune pool diversity and even only a few subclones. The diversity of the immune repertoire is influenced by individual exposure to specific pathogen antigens, and patients' health should be carefully assessed in studies. The maturation and advancement of high-throughput sequencing technologies and methods provides new opportunities to study the immune pool characteristics of NMOSD patients. However, it should be recognized that high-throughput sequencing technologies are still relatively expensive, the amount of data generated is huge, and the process of data interpretation and analysis is complex, and existing clinical studies are limited by the number of samples. Therefore, the clinical application of immune pools requires the study of hardware and software and a large amount of data. Applying immunomic libraries in a clinical setting requires exploration and collection of hardware, software, and large amounts of data. Although this study is limited by the number of cases, if the number of cases is expanded and the findings are confirmed in more studies, it is expected to provide new important clinical monitoring indicators for the diagnosis, treatment, and evaluation of NMOSD diseases. Further understanding of the characteristics of the BCRIgH-CDR3 gene can provide a further understanding of the occurrence, development, and immune response mechanism of NMOSD, thereby laying the foundation for the immunotherapy and clinical application of NMOSD.

## Figures and Tables

**Figure 1:** Schematic diagram of neuron structure.

**Figure 2:** Schematic diagram of the basic structure of the neural network.

**Figure 3:** Length distribution of IgG-CDR3 amino acid sequences in peripheral blood B cells.

**Figure 4:** Frequency distribution of TOP20-V and J genes.

**Figure 5:** ROC curve analysis of Rello signal in AQP4 antibody-positive patients and healthy controls.

**Figure 6:** ROC curve analysis of Relo signal in MOG antibody-positive optic neuritis patients and healthy controls.

**Figure 7:** ROC curve analysis of Relo signal in both patients and healthy controls.

**Figure 8:** Correlation analysis between serum IL-36 levels and clinical characteristics in NMOSD patients.

**Figure 9:** Correlation analysis between serum IL-36 level and the number of involved spinal cord segments.

**Figure 10:** Correlation analysis between serum IL-36 level and EDSS score.

**Table 1:** Basic information of immune repertoire of research specimens.

	Sample	Age	Hormone dosage (mg)	CDR3read count	CDR3 types	Types of CDR3/number of CDR3reads
Early treatment	Patient 1	38	500	4119645	15342	0.0054
	Patient 2	35	1000	2490645	16423	0.0034
	Patient 3	38	1000	3634664	211534	0.0043
	Patient 4	32	80	2859455	11953	0.0045
	Patient 5	33	80	286864	11254	0.0037
	Patient 6	44	500	3564265	11445	0.0033

Stable period	Patient 1	45	10	37 55562	11312	0.0031
	Patient 2	36	20	3836250	19721	0.0052
	Patient 3	34	20	2665460	8832	0.0033
	Patient 4	33	10	3064539	13021	0.0043
	Patient 5	33	5	2854535	8713	0.0036
	Patient 6	44	5	3563451	16987	0.0045

Normal control	NO01	34	—	4062532	20186	0.0052
	NO02	35	—	3332535	11043	0.0034
	NO03	36	—	2843250	11984	0.0044
	NO05	47	—	3353432	14242	0.0046
	NO07	46	—	3853421	22435	0.0054
	NO08	35	—	3483240	13324	0.0035


**Table 2:** Statistics of clonal diversity indicators.

	Sample	Clone	ChaoE	Chao1	Shannon Wiener Index	Inverse Simpson Index	D50
Early treatment	Patient 1	15322	15756	32343	7.5545	1484.43	3.64
	Patient 2	16435	22325	43545	8.0534	2541.42	5.93
	Patient 3	21345	22321	48436	8.2033	2905.85	5.3
	Patient 4	11123	15214	31633	7.3734	1290.42	4.09
	Patient 5	11212	14342	31563	7.0335	921.833	3.15
	Patient 6	11434	12423	29546	6.7953	730.21	2.44

Stable period	Patient 1	11425	12023	26943	6.7835	714.92	2.37
	Patient 2	19231	20343	46543	7.865	2125.32	4.163
	Patient 3	8834	12324	27446	6.635	680.31	3.93
	Patient 4	13042	15843	33345	7.3834	1342.81	0.63
	Patient 5	8753	11524	38535	5.1435	138.24	4.69
	Patient 6	16432	17923	43455	7.8653	2013.23	4.23

Normal control	NO01	20132	20324	28145	7.9654	2263.42	3.78
	NO02	11434	13643	30656	7.2445	1113.23	4.18
	NO03	11433	15344	39164	7.3954	1323.74	4.63
	NO05	14343	16434	49467	7.7245	1825.43	4.63
	NO07	22234	23145	34357	8.1045	2708.43	4.37
	NO08	13349	14844	32787	7.4954	1521.43	3.64


**Table 3:** Two lgH-CDR3-dominant sequences in the early treatment group of NMOSD patients.

v	d	j	Frequency of early treatment group in NMOSD patients					
			Patient 1	Patient 2	Patient 3	Patient 4	Patient 5	Patient 6
IGHV1-3	IGHD6-19	IGHJ6	1913	6	1167	4590	7430	6323
IGHV5-51	IGHD3-10	IGHJ6	4	1573	3	2	1791	3136

**Table 4:** Two kinds of lgH-CDR3-dominant sequences of NMOSD patients in stable treatment group.

v	d	j	Frequency of early treatment group in NMOSD patients					
			Patient 1	Patient 2	Patient 3	Patient 4	Patient 5	Patient 6
IGHV1-3	IGHD6-19	IGHJ6	1889	6	0	1324	4	6
IGHV5-51	IGHD3-10	IGHJ6	2	0	6	2	1	8

## Data Availability

No data were used to support this study.
